The article "Analysis of China's Population Flow between Urban and Rural Areas and the Reform of Public Health Old-Age Insurance System under the Background of Sustainable Ecological Environment" was retracted in 2023. Reason: compromised peer review.

# Analysis of China's Population Flow between Urban and Rural Areas and the Reform of Public Health Old-Age Insurance System under the Background of Sustainable Ecological Environment

**DOI:** 10.1155/2022/9752913

**Published:** 2022-06-22

**Authors:** Hailiang Guo, Qiangqiang Luo

**Affiliations:** ^1^School of Law, Ningxia University, Yinchuan 750021, Ningxia, China; ^2^School of Government, Yunnan University, Kunming 6500091, Yunnan, China

## Abstract

The future impact of population development trend on social security is extremely huge and far-reaching, to conform to the law of population mobility to adjust the relevant policies, this study is for the urban and rural flow of the Chinese population, and the public health endowment insurance system analyzes the implementation status of PHEI of China's floating population and the existing problems of labor dispatch and employee endowment insurance system. Questionnaires were distributed to 3000 high-quality migrant workers who participated in the training of high-quality migrant workers in 6 cities in Central China where labor export is concentrated and 1000 fresh graduates from agricultural colleges and universities; through the bivariate *t*-check model in SPSS software, this study analyzes the needs of landless farmers, agricultural scientific and technological talents, and employed people for the living environment. The results show that from the population outflow and population inflow process there has been certain influence on the sustainable ecological environment; this study puts forward the reform of public health endowment insurance system of floating population, the strategy means in accelerating the rural talent revitalization, for the sustainable development of rural areas that has a significant positive effect.

## 1. Introduction

Since the 1980s, China's population flow has gradually increased. On February 23, 2021, the general office of the CPC Central Committee and the general office of the State Council issued the opinions on accelerating the revitalization of rural talents and asked all localities to study and implement them [1]. The document points out that “the key to rural revitalization lies in people.” It should be made use of public service facilities such as high-quality migrant workers' skill training institutions and labor dispatch agencies established by governments at all levels to improve the knowledge and skill quality of migrant workers and strengthen the comprehensive service to the floating population [2]. On the other hand, the document requires professional and technical talents to go deep into the field and “write papers on the Earth” and solve the problem of public health and old-age insurance after professional and technical talents go to the countryside [3]. After professional and technical personnel go deep into the countryside, they will bring technical support to the water and soil environment management, mountain forest and windbreak forest management, and the optimization and regulation of farmland and water conservancy facilities in rural areas, effectively improve the ecological environment in rural areas, and realize the sustainable development of rural areas.

Li studied the actual value of the floating population in first-tier cities from the contribution of the floating population community construction in the place where the floating population is imported. When most cities treated the consequences of the floating population input as a persistent social disease, the study pointed out that the inflow process of the floating population is of positive significance to the urban community construction [4]. Yang et al. pointed out in their research that the completeness of urban infrastructure and urban ecological environment directly affects the attraction of cities to the floating population. Perfect urban infrastructure and ecological environment protection of urban circle can effectively promote the input enthusiasm of the floating population [5]. The above two research results focus on the attraction of big cities to the floating population. Their common opinion is that the ecological environment of cities directly improves the attraction of cities to floating population, and the consequences of floating population entering cities, although it will bring some pressure to urban infrastructure, can also promote urban construction and development. Ma et al. put forward the collaborative development model of “industry population ecology.” This study takes the population inflow of the Fujian tea industry as an example to explore the feasibility of attracting talent inflow after the development of rural industrialization [6]. Zhang et al. also discussed the attraction of rural industrialization to talents outside the region by taking the talent introduction in rural areas of Anhui Province as an example. Traditional Chinese medicine planting enterprises, agricultural product deep-processing enterprises, and forestry planting and particle board processing enterprises in Anhui have attracted high-quality talents [7]. That is, the way for rural areas to attract external talents with high academic qualifications, high professional titles, and high quality is to form agricultural production businesses into enterprises above the designated scale and attract relevant talents with agricultural enterprises. Xian pointed out that the aging trend of the society is increasingly serious, and the number of empty nesters and left-behind elderly under the influence of the urbanization trend is increasing, which hides the huge pressure on social pension. Therefore, how to implement the living security of the elderly and public health medical security is the top priority to achieve elderly care [8]. According to Li et al., the rise of cities is often accompanied by large-scale population flow, as the new generation of floating population has a profound impact on the social and urban economic development. Regarding the social integration of the new generation of population, it is conducive to attracting the inflow of young floating population in various regions and is of great significance to promoting the improvement of economic and employment structure and giving play to the positive role of population mobility [9].

This study will explore the impact of population flow between urban and rural areas and public health endowment insurance on the sustainable ecological environment in two aspects: the impact of population outflow process and population inflow process on the sustainable ecological environment.

## 2. Implementation Status of Public Health Endowment Insurance for China's Floating Population

### 2.1. Implementation Status of Endowment Insurance for High-Quality Migrant Workers

High-quality migrant workers are defined as those who have intermediate or high school (some skill certificates require a college or bachelor's degree or above), participated in the training of new professional farmers, obtained the training certificate, issued the certificate by the county-level new professional farmers, and hold the land-lost farmers with skill certificates issued by the relevant ministries and commissions or industry associations (associations) [10]. In order to improve the income level of the rural population, the state provides full or even excess subsidies for the training process of relevant certificates. At the same time, each township organization connects with the construction site and entrusts the labor dispatch company to carry out the collective labor dispatch work. Together with labor dispatch companies, township governments provide high-quality migrant workers with wage advances, social security withholding, collective rights protection, and other services [11].

The migrant workers registered residence in the four forms of social insurance. First, agricultural household members can participate in rural cooperative social insurance in the rural areas and communities where the registered residence is located. Second, the urban household registration personnel can participate in the cooperative social insurance of the urban residents in the community where the household register is located. In addition, the high-quality migrant workers participate in the social insurance for the employees of the enterprises, and they can choose to handle relevant social security accounts at the site. Relevant social security accounts can also be handled at the place of dispatch [12]. According to the statistical information released by the official website of the Ministry of Human Resources and Social Security, among all the floating population participating in social insurance, the selection results of various social insurance organization forms are shown in Figure 1.

In Figure 1, the rural cooperative social insurance accounts for 52%, the urban cooperative social insurance accounts for 23%, and the sum of the two accounts for 75%. These two models are counted as freelancers or unemployed by the Ministry of Human Resources and Social Security. This model has become the main form for high-quality migrant workers to choose social insurance. Migrant workers registered residence in the registered residence of 18% of the staff members of the social insurance office, and the social insurance payment is only 7% of the household social insurance coverage. That is, high-quality migrant workers are unwilling to choose the workers' social insurance paid by the labor dispatching agencies in the registered residence area. The fundamental reason is that the partial withholding base of their medical insurance is relatively high and the reimbursement ratio is low.

### 2.2. Implementation Status of Endowment Insurance for the Introduction of Rural Technical Talents

According to the opinions on the revitalization of rural talents, all localities, under the strong supervision and strong subsidies of the government, introduce highly educated talents in agriculture, forestry, animal husbandry, aquaculture, veterinary medicine, food, agricultural finance, agricultural supply chain, and other fields, generally those with bachelor's degree or above, with certain agricultural project management experience and can work on the construction site for a long time [13].

At present, the coverage of endowment insurance is not high, and there is still a lot of room for improvement. Because the publicity is not in place, farmers keep the new farmers in a certain misunderstanding, and the subsidy level is also low, leading to the low enthusiasm of farmers to participate in the insurance, so we should steadily improve the important support of endowment insurance through the way of subsidies. In the same way, the above four forms of social insurance organizations are investigated. In the statistical information published on the official website of the Ministry of Human Resources and Social Security, the composition of social insurance when introducing technical talents in rural areas is shown in Figure 2:

Figure 2 shows city registered residence in the city of talent introduction, the social insurance organization for the employees in the rural area is about 49%, and the other social insurance organizations are the social security for workers in the household registration area (about 38%) and the registered residence free occupation social insurance (about 13%). Registered residence occupation social insurance comes from the social insurance of professional and technical personnel dispatched by the professional and technical personnel in the process of enterprise university research cooperation, while the registered residence freelance social insurance comes from the social insurance of the agricultural-related free engineer studio or the agricultural senior manager studio. The social insurance for site employees comes from the social insurance paid by professional and technical talents who directly handle the contract system.

## 3. Labor Dispatch and Existing Problems of Employee Pension Insurance System

### 3.1. Compliance with Labor Dispatch

An internet company's survey on the collective labor dispatch under the high-quality migrant workers project found that more than half of the high-quality migrant workers did not participate in the labor dispatch but chose to find their own jobs. Among the high-quality migrant workers participating in the collective labor dispatch, more than six pairs expressed dissatisfaction with the dispatch process. The current collective labor dispatch system of migrant workers with high quality does not fully meet the current collective needs of migrant workers. The study will conduct an independent investigation based on the survey results to find relevant problems.

Labor dispatch should inform the exchange of company basic situation and explain, understand the actual working environment, jobs, if necessary to investigate, for the greatest interests of migrant workers, and the most important point is to stand on the intention of consider sending, confirm suitable for the type of work, respect the choice of migrant workers, according to the needs and standards of choosing and employing persons to arrange work, and ensure labor dispatch compliance strategy.

### 3.2. Enthusiasm for Rural Talent Introduction

The main institutions for the introduction of rural talents are planting and breeding agricultural enterprises and food processing enterprises in rural areas. These enterprises have small-scale and thin profits. If highly educated and high-quality technical talents are employed, although it can bring technological upgrading, it will also bring pressure on the cost of human resources [14]. Therefore, the enthusiasm of most small and microagricultural enterprises to introduce technical talents is not high. At the level of technical talents, because participating in the introduction project of technical talents requires stable employment in rural areas, these high-quality and highly educated talents need to leave the first- and second-tier cities with superior living environment and enter rural areas, so their personal enthusiasm is also low. Therefore, there are serious problems in the implementation path of the rural talent introduction process, resulting in low enthusiasm on both sides and low efficiency of project promotion.

## 4. Social Investigation and Analysis of People's Needs

### 4.1. Implementation Plan of Social Investigation

Through the network questionnaire method, a questionnaire was distributed to 3000 high-quality migrant workers participating in the training of high-quality migrant workers in six cities in Central China where labor export is concentrated. The respondents were asked to choose 1–5 levels from all descriptions, corresponding to 1–5 points in the statistical results.

Through the network questionnaire method, a questionnaire was distributed to 1000 fresh graduates from agricultural undergraduate colleges and universities, and questions and answers were put forward on the above two questions and environmental protection-related questions. Respondents were required to select 5 levels from 1–5 of all descriptions, corresponding to 1–5 points in the statistical results.

The data comparison method adopts the mode of bivariate *t*-check in SPSS software, and the calculation method is shown in formula (1)as follows:

(1) $$\begin{array}{c} t=\frac{\mu_{1}-\mu_{2}}{\sqrt{\left(\left(n_{1}-1\right)s_{1}^{2}+\left(n_{2}-1\right)s_{2}^{2}\right)/\left(n_{1}+n_{2}-2\right)\left(\left(1/n_{1}\right)+\left(1/n_{2}\right)\right)}}. \end{array}$$

Among them, *μ*_1_, *μ*_2_ is the arithmetic mean of sequence 1 and sequence 2. The calculation method is as follows in formula (2); *n*_1_, *n*_2_ is the number of elements in sequence 1 and sequence 2; *s*_1_, *s*_2_ is the standard deviation rate of sequence 1 and sequence 2; and the calculation formula is shown in formula (3) below.

(2) $$\begin{array}{c} \mu =\frac{1}{n}\sum_{i=1}^{n}x_{i}. \end{array}$$

Among them, *x*_*i*_ is the ith measured value in the sequence; *N* is the number of elements in the sequence, corresponding to *n*_1_, *n*_2_ in formula (1) above; and *μ* is the calculation result of arithmetic mean, corresponding to *μ*_1_, *μ*_2_ in formula (1) above

(3) $$\begin{array}{c} s=\frac{1}{n-1}\sqrt{\overset{n}{\underset{i=1}{\sum }}{\left(x_{i}-\mu \right)}^{2}.} \end{array}$$

Among them, the meaning of mathematical symbols is the same as formula (1) and formula (2) above; the smaller the *t* value obtained from the two columns of data, the greater the difference between the data. From the range of *t* value, when *t* < 10.000, it is considered that the data are statistically different; on the contrary, it is considered that the data are statistically consistent. SPSS built-in algorithm is used to calculate the reliability *p* value of synchronous output when *t* value is obtained. When *p* < 0.05, it is considered that the statistical result is statistically significant. When *p* < 0.01, it is considered that the statistical result is statistically significant. The smaller the *p* value, the higher the data reliability.

### 4.2. Demand Analysis of Landless Farmers

Considering the age-group of migrant workers, the questionnaire survey results of landless farmers participating in high-quality migrant workers' project are shown in Tables 1 and 2:

In Table 1, people aged 25 to 35 years are more likely to choose independent employment, while those under 25 years old are more dependent on labor dispatch, and those over 36 years old are more dependent on labor dispatch. All data have *t* < 10.000, *p* < 0.05, with a credible statistical difference, while the statistical results of people under 35 years old have *t* < 10.000, *p* < 0.01, with a significant statistical difference. That is, the current promotion of high-quality migrant workers' project, including skill training subsidies for migrant workers and collective labor dispatch, focuses more on young migrant workers under the age of 25 years.

In Table 2, as the age of migrant workers increases, their intention to participate in local employment also gradually increases, and their intention to go to other places for employment continues to weaken.

### 4.3. Demand Analysis of Agricultural Scientific and Technological Talents

Considering the academic grouping of agricultural scientific and technological talents, the questionnaire survey results for agricultural scientific and technological talents are shown in Tables 3 and 4:

In Table 3, all data have *t* < 10.000, *p* < 0.01, with a significant statistical difference. According to the data, only 22.5% to 27.8% of agricultural college graduates hope to work in frontline units of agricultural production, while agricultural college graduates focus more on going to small and medium-sized cities to engage in teachers, civil servants, and other occupations, and agricultural college graduates focus more on going to core big cities to engage in it, e-commerce, finance, and other occupations. Therefore, although there are more than 10000 agricultural graduates in colleges and universities every year, fewer graduates can actually participate in the construction of the front line of agricultural production. By analyzing the employment intention of graduates willing to go to the front line of agricultural production, Table 4 is obtained.

In Table 4, all data have *t* < 10.000, *p* < 0.01, with a significant statistical difference. The data show that the employment intention of large-scale agricultural enterprises is weak, followed by ecological agricultural enterprises. Most large-scale agricultural enterprises are central enterprises or listed enterprises, and the entry threshold is high, so most agricultural college graduates quit in the face of difficulties. Ecological agricultural enterprises are generally small in scale and are mostly combined with new sales models. They generally adopt the full-time sales management model, and the enterprise stability and poststability are low. Therefore, it is difficult for graduates to adapt. In order to make it easier to observe the data, the data in Table 4 above are visualized to get Figure 3.

In Figure 3, the three agricultural production frontline employment directions with the highest employment intention are agricultural tourism integrated enterprises, with a total employment intention of 66.5%, followed by agricultural product supply chain or agricultural finance enterprises, with a total employment intention of 58.6%, and then agricultural processing integrated enterprises, with a total employment intention of 46.3%. It can be found that graduates of this college pay more attention to the stability of work and after when they choose jobs in the front line of agricultural production.

### 4.4. Demand Analysis of Employed Persons for Living Environment

The environmental factors should be investigated that may affect the employment direction of the floating population (including migrant workers and agricultural professional and technical talents), including regional climate, air quality, transportation convenience, perfection of medical and educational facilities, and wage level (calculated by the ratio of annual salary-to-house price). The comprehensive statistical results of relevant questions are shown in Table 5:

In Table 5, with the increase in educational background, the employment city choice intention of the relevant floating population has a linear change trend. For example, with the increase in educational background, the demand for climate and air quality and educational supporting facilities increases, while the demand for transportation convenience, wage level, and medical supporting facilities decreases. In order to more intuitively observe the above data, the above data should be visualized to obtain Figure 4.

In Figure 4, the main demand of all floating population flowing into the city comes from the ratio of annual salary-to-house price (wage level) of the city. If the per capita annual salary is an economic index and it is difficult to adjust in the short term, the local government should reasonably control the house price and improve the ratio of annual salary to the house price, which will effectively enhance the attraction of the city to the floating population. In particular, if local governments want to choose the return of migrant workers to promote the large-scale development of local agricultural industrialization, they should carry out urban environmental infrastructure from the abovementioned annual salary-to-house price ratio, medical facilities, and transportation convenience. If they want to attract highly educated agricultural talents, they should carry out urban environmental construction from the aspects of education facilities and ecological environment governance. It can be considered that the construction of a sustainable urban ecological environment includes not only natural ecological problems such as climate and air quality but also many economic, geographical, and ecological problems.

## 5. Reform Strategy of Public Health Endowment Insurance System for Floating Population in China

### 5.1. Labor Dispatch System Should be Transformed into Labor Service System

In the social survey, it is found that migrant workers' guidance and coordination of labor export work are aimed at large enterprises. On a better working platform, seeking the impact of the establishment of labor cooperation and labor dispatch system on the labor service system and actively exploring ways to solve the impact can effectively mobilize the enthusiasm of workers' dispatch work, safeguard the interests of migrant workers, and reduce the resistance of migrant workers. Moreover, the direction of collective labor dispatch is mostly miscellaneous workers on the construction site and general workers on the production line, and few can be dispatched to the professional skills' counterpart positions of high-quality migrant workers, which exacerbates the resistance of migrant workers to collective labor dispatch.

Observing the process of collective labor dispatch from the government side, we will find that the government mainly has two needs: one is to maintain the stability of landless farmers through collective labor dispatch, and the other is to realize the local collection and payment of individual income tax and surtax through collective labor dispatch. If the process is completely handed over to enterprises, and the government only promotes collective labor dispatch from the aspect of intergovernmental docking, the above disadvantages will be avoided to a certain extent. Most migrant workers trust their village foremen to lead the team to find jobs. The government can encourage such foremen to establish formal enterprises, standardize their operations, and give subsidies to labor dispatch companies to these village-run enterprises.

The social environment is an important part in the process of sustainable environmental control. The government should go deeper into the grassroots level in relevant work, do a good job in grassroots research, and continuously improve the work process, so as to truly realize the stability maintenance of landless farmers through the high-quality migrant workers' project.

### 5.2. The Construction of Urban Ecological Environment Has a Direct Effect on the Attraction of Floating Population

The urban ecological environment includes not only the natural environment but also the economic and geographical environment of the city. For example, urban infrastructure construction, urban public transport, and intercity transportation systems need to be continuously improved, urban education and medical supporting systems need to be continuously constructed, and urban living material support capacity also needs to be invested. If the urban economic and geographical environment cannot be synchronized with the natural environment, it is difficult to effectively control the return of migrant workers and let alone effectively attract the inflow of high-quality and highly educated talents.

The trend of population flow in rural areas is mainly reflected in two points: one is that landless farmers with low educational level flow out of rural areas; the other is that highly educated and high-quality talents enter agricultural enterprises for employment, and private capital continues to flow into rural areas for investment. Over the past five years, agriculture has developed into a blue ocean industry, with a significantly higher return on investment than other industries, but the investment risk is also high. The traditional farmers under the small-scale peasant economic model are difficult to make profits in the new countryside, and the small-scale peasant thought is difficult to bear such a large investment risk, so this exchange population flow appears.

However, the infrastructure level in rural areas is poor, the ability of living security is not strong, and the economic and geographical environment is relatively bad. It will be more difficult to allow high-quality talents to flow to rural areas. In the new rural construction, we should focus on rural infrastructure, and the infrastructure process should not damage the rural natural environment. This puts forward higher requirements for the level of urban infrastructure planning.

### 5.3. The Inflow of Floating Population Can Effectively Improve the Local Urban Ecological Environment

Relevant studies have pointed out that for the first- and second-tier cities, the inflow process of migrant workers can effectively promote the basic service capacity of cities and effectively increase grassroots labor resources. For rural areas, the inflow of high-quality and highly educated talents can effectively improve the local economic and industrial management level, bring new development power to the local rural infrastructure, and effectively improve the local level of urban-rural integration.

Taking large-scale agricultural enterprises, integrated agricultural processing enterprises, and integrated agricultural tourism enterprises as examples, due to the addition of high-quality talents, the agricultural production and management level of enterprises can be effectively improved, the land output rate can be increased, the utilization rate of water and soil can be increased, and the sustainable development ability of cultivated land can be increased. Furthermore, the participation of high-quality talents can effectively combine agricultural production with environmentally sustainable development.

However, this principle will bring a strange circle to the agricultural underdeveloped areas, that is, because the local new agricultural development level is low, it is difficult to introduce a high-quality floating population, and with the lack of a high-quality floating population, the local new agricultural development is difficult to sustain. Therefore, the government in the underdeveloped areas of new agriculture should take the investment attraction of new agriculture as the key investment attraction direction and obtain the initial development power of local new agriculture by introducing new agricultural operation enterprises above foreign scale.

## Figures and Tables

**Figure 1:** Social insurance organization form of high-quality migrant workers.

**Figure 2:** Social insurance organization form of introducing technical talents in rural areas.

**Figure 3:** Distribution of intention of agricultural college graduates to go to the front line of agricultural production.

**Figure 4:** Statistical chart of demand for the living environment of employed persons.

**Table 1:** Distribution map of employment mode intention of landless farmers of different ages (%).

Grouping	<25	25–35	>36	Total
Independent employment	34.7	72.8	45.4	58.3
Dispatch employment	65.2	27.2	54.6	41.7
*t*	2.276	2.189	6.742	7.295
*p*	0.008	0.007	0.016	0.019

**Table 2:** Distribution map of employment intention of land-lost farmers of different ages (%).

Grouping	<25	25–35	>36	Total
Local employment	28.5	39.2	57.4	51.1
Foreign employment	71.5	60.8	42.6	48.9
*t*	1.052	3.713	8.149	12.501
*p*	0.002	0.006	0.009	0.012

**Table 3:** Distribution map of employment intention of agricultural scientific and technological talents (%).

	Specialty	Undergraduate	*t*	*p*
Core city circle	36.2	38.6	7.292	0.006
Small city	41.3	33.6	5.307	0.005
Front line of agriculture	22.5	27.8	6.247	0.007

**Table 4:** Distribution map of employment intention of agricultural scientific and technological talents in the front line of agricultural production (%).

	Specialty	Undergraduate	*t*	*p*
Scale agriculture	3.6	3.1	6.792	0.005
Agricultural processing integration	24.7	21.6	8.925	0.009
Agricultural tourism integration	35.2	31.3	8.131	0.008
Ecological agriculture	12.4	9.4	5.294	0.006
Supply chain or commerce	24.1	34.6	1.083	0.001

**Table 5:** Demand for the living environment of employed persons.

	Migrant worker	Agricultural junior college	Undergraduate course in agriculture
Climate	1.6	2.2	5.5
Air quality	2.8	2.9	5.7
Convenient transportation	23.6	21.8	19.8
Medical facilities	12.5	12.3	11.9
Education supporting	3.2	17.5	24.4
The wage level	56.3	43.3	32.7

## Data Availability

The data underlying the results presented in the study are available within the article.
